The article "Construction of a Fundamental Quantitative Evaluation Model of the A-Share Listed Companies Based on the BP Neural Network" was published in 2022. Journal: Comput Intell Neurosci.

# Construction of a Fundamental Quantitative Evaluation Model of the A-Share Listed Companies Based on the BP Neural Network

**DOI:** 10.1155/2022/7069788

**Published:** 2022-03-01

**Authors:** Yankai Sheng, Kui Fu, Jing Liang

**Affiliations:** School of Economics, Wuhan University of Technology, Wuhan 430070, China

## Abstract

Quantitative investment has attracted much attention, along with the vigorous development of Fintech. Fundamentals are one of the most important reference factors for investment. Before quantitative trading, evaluation of fundamentals may have been more dependent on personal experience. While artificial intelligence evaluation models can provide good investment suggestions and select stocks with better fundamentals. From the four angles of solvency, growth ability, operation ability, and profitability, this research selects 13 financial indicators to build a fundamental evaluation system through correlation coefficient analysis. The corporate life cycle assessment indicator is innovatively added so that the fundamental improvement expectation is put into the evaluation system. Four different kinds of scoring methods are applied to obtain a more rational and comprehensive evaluation of indicators. Then, grey relational analysis is adopted to determine the initial weight to calculate the expected output. Finally, BP neural network (back propagation) is used for training and testing to realize weight optimization. It is concluded that the model is suitable for quantitative scoring of the fundamentals of listed companies and can effectively reflect their value of them.

## 1. Introduction

Since Benjamin Graham founded the theory of value investment [1], the fundamentals of stocks have become an indispensable factor of investment. A large number of econometric models used to evaluate the intrinsic value of companies have emerged, such as Tobin's Q theory [2, 3] and five-factor asset pricing model [4], which pushed the development of value investment. However, traditional econometric models are limited due to a lack of proof to demonstrate that the result is optimal.

With the blossom of FinTech and quantitative investment, artificial intelligence algorithms are widely used to optimize the results of traditional models and construct better portfolios. For example, a classifier model called SVM (support vector machines) has been shown to perform well in stock price forecasting [5] and financial distress [6]. Moreover, researchers have conducted a vast investigation on artificial neural networks used in the financial field such as BP (back propagation) neural network [7], LSTM (long short-term memory) neural network [8], and NARX (nonlinear autoregression exogenous) neural network [9].

The article "Construction of a Fundamental Quantitative Evaluation Model of the A-Share Listed Companies Based on the BP Neural Network" was published in 2022. Journal: Comput Intell Neurosci.

Motivated by the above observations, this paper focuses on the construction of a fundamental quantitative evaluation model of the A-share listed companies based on the BP neural network. In section 2, the theoretical basis of the model is provided, in order to explain the background concepts and related technologies. In section 3, this paper provides the detailed process of model construction, including the determination of expected output and parameter setting. In section 4, the results of the model are analyzed. In section 5, the conclusion and outlook are summarized.

The contribution of this research can be concluded as follows:

1. When the indicator is under a dimensionless process, a variety of evaluation methods are innovatively combined, so that the indicator score is more reasonable and comprehensive.
2. With the corporate life cycle evaluation indicator added, the companies with fundamental improvement expectations can be identified. Since the cash flow statement is included in the evaluation system, all the important data from the three statements are included in the evaluation model for the first time.
3. Grey relational analysis and BP neural network training simulation are used to optimize the weight of indicators so as to obtain the fundamental scoring system of all-industry listed companies.

## 2. Theoretical Basis of Model Construction

### 2.1. Grey Relational Analysis

Grey relational analysis is a quantitative description and comparison of the development state of objects so as to analyze and determine the influence degree between the contribution measure of factors on the main behavior. The Grey correlation degree is a measure of the correlation between two systems. If the relative change situation of the two factors is consistent in the development process, the grey correlation degree of the two factors is large; otherwise, it is small. Grey relational analysis is usually used to address the comprehensive evaluation problem [10]. Chen et al. [11] evaluated the growth of small and medium-sized listed companies through grey relational analysis, and concluded that the obtained information can be fully used with this method; Zhang et al. [12] established a quantitative evaluation model of strategic emerging industries through grey relational analysis, which made the evaluation system more reasonable; Delcea et al. [13] put forward suggestions on corporate development and extreme situation response by using the quantitative results obtained with grey relational analysis. Therefore, it is concluded that grey relational analysis is suitable for quantitative scoring of the fundamentals of listed companies, and it is reasonable to take it as the expected output of the BP neural network. The progress of grey relational analysis is shown as follows:

**Step 1 .**

: The data after standardization is used to gain the grey correlation degree coefficients *ζ*_*i*_(*k*) of the reference series and comparison series with formula (1).

(1) $$\begin{array}{c} \zeta_{i}\left(k\right)=\frac{\underset{i}{\min}\underset{k}{\min}\left|g_{0}\left(k\right)-g_{i}\left(k\right)\right|+\rho \underset{i}{\max}\underset{k}{\max}\left|g_{0}\left(k\right)-g_{i}\left(k\right)\right|}{\left|g_{0}\left(k\right)-g_{i}\left(k\right)\right|+\rho \underset{i}{\max}\underset{k}{\max}\left|g_{0}\left(k\right)-g_{i}\left(k\right)\right|}. \end{array}$$

In formula (1), *g*_*i*_(*k*) is the score of indicators of listed companies and *ρ* is the resolution coefficient. The usual practice is adopted in this paper where *ρ*  = 0.5.

The article "Construction of a Fundamental Quantitative Evaluation Model of the A-Share Listed Companies Based on the BP Neural Network" was published in 2022. Journal: Comput Intell Neurosci.

**Step 2 .**

: When the calculated grey relational degree coefficient is obtained, the weight calculation formula is used to obtain the weight of the indicators.

(2) $$\begin{array}{c} \omega_{i}=\frac{\sum_{k=1}^{n}g_{i}\left(k\right)}{\sum_{k=1}^{n}\sum_{i=1}^{m}g_{i}\left(k\right)}. \end{array}$$

In formula (2), *n* is the number of sample companies and *m* is the number of selected indicators.

**Step 3 .**

: According to the weights gained, the scores of listed companies are calculated by formula (3) as the expected output of the neural network model.

(3) $$\begin{array}{c} G\left(k\right)=\overset{m}{\underset{i=1}{\sum }}\omega_{i}\cdot g_{i}\left(k\right). \end{array}$$

In the formula, *G*(*k*) means the score of the company.

### 2.2. BP Neural Network

The BP (back propagation) neural network, proposed by scientists led by Rumelhart and McClelland in 1986, is a gradient descent method, being able to optimize the weight and threshold through error[14]. Zhang Xuemin et al. [15] have combined an analytic hierarchy process and BP neural network to build an early warning evaluation system in order to keep poverty-stricken people from returning to poverty in specific areas; Zhang Zhengang et al. [16] used information entropy theory to determine the index weight and then used BP neural network training and simulation to construct the performance evaluation system of listed white household appliances companies in China. Thanks to its advantages in weight optimization, the BP neural network can be effectively applied to the weight selection of the quantitative evaluation system constructed in this paper. The structure of the BP neural network is shown in Figure 1.


(6) $$\begin{array}{c} \Delta w_{ij}=-\eta \frac{\partial Error}{\partial w_{ij}}\text{i}=1\text{,}2\text{,}...\text{,m, j}=1\text{,}2\text{,}...\text{,n.} \end{array}$$

(7) $$\begin{array}{c} \Delta v_{jk}=-\eta \frac{\partial Error}{\partial v_{jk}}\text{k}=1\text{,}2\text{,}...\text{,n, j}=1\text{,}2\text{,}...\text{,n.} \end{array}$$

A routine BP neural network has 3 layers: input layer, hidden layer, and output layer. In Figure 1, *x* is the input data, and *y* is the output data. Assume the weight of neurons in the hidden layer is *w*, and the weight of neurons in the output layer is *v*. Assume *d* is the expected output, then the error of the model *Error* can be defined by formula (4) as follows:

(4) $$\begin{array}{c} Error=\frac{1}{2}\overset{n}{\underset{k=1}{\sum }}{\left(d_{k}-y_{k}\right)}^{2}. \end{array}$$

In formula (4), *y*_*k*_ can be denoted by formula (5), where *f* is the activation function.

(5) $$\begin{array}{c} y_{k}=f\left(\overset{n}{\underset{j=1}{\sum }}v_{jk}f\left(\overset{m}{\underset{i=1}{\sum }}w_{ij}x_{i}\right)\right). \end{array}$$

If *Error* does not reach the target, the neural network will adjust *w* and *v*. The adjustment amount Δ*w*_*ij*_ and Δ*v*_*jk*_ are defined by formula (6) and formula (7), where *η* is learning rate.

The article "Construction of a Fundamental Quantitative Evaluation Model of the A-Share Listed Companies Based on the BP Neural Network" was published in 2022. Journal: Comput Intell Neurosci.

After the neural network calculates for a certain time until the *Error* reaches the target, the iteration will stop.

### 2.3. Corporate Life Cycle Theory

As early as the 1950s, Mason et al. [17] put forward that the development stage of a company can be viewed from the perspective of its life cycle. Since then, researchers have proposed a large number of life cycle stage division models, which are mainly based on the accounting indicators related to corporate organizational behavior and corporate value, where the life stages of a company are divided into segments from 3 to 10 [18]. The purpose of this paper is to establish a quantitative model so as to find a suitable method from the perspective of corporate accounting indicators. Ye [19] has put forward a revised model of the corporate life cycle based on sales and divided the corporate development into four stages. Zhang et al. [20] used the main business income growth rate, retained yield, capital expenditure rate, corporate age, and other indicators to divide the corporate life cycle and analyze its impact on the overinvestment of the company. Cao et al. [21] divided the corporate development stages into the initial stage, growth stage, maturity stage, and recession stage with the method of combination of cash flow components and discussed the corporate financial distress in different development stages, respectively.

Being the most widely used method, the cash flow combination method divides the development of companies into four stages: the start-up stage, the growth stage, the mature stage, and the recession stage, which is the method used in this paper. The division is based on Table 1.

The article "Construction of a Fundamental Quantitative Evaluation Model of the A-Share Listed Companies Based on the BP Neural Network" was published in 2022. Journal: Comput Intell Neurosci.

## 3. Model Construction

### 3.1. Selection of Indicators

Referring to the research of Yao Hui and Zhang Hu et al. [20,21,22], 14 indicators are selected for analysis from four dimensions as shown in Table 2: solvency, growth ability, operation ability, and profitability, as well as corporate life cycle judgment.

### 3.2. Selection of Evaluation Methods

According to the characteristics of different indicators, different evaluation methods are selected to turn raw data into a dimensionless score.

#### 3.2.1. Standardized Evaluation

The indicators are standardized by formula (8) to map the data to the interval of [0, 100] to complete the scoring of a single index directly. Standardization evaluation consists of forward standardization evaluation and inverse standardization evaluation, shown as follows:

(8) $$\begin{array}{c} g=\frac{x-\text{min}\left(X\right)}{\text{max}\left(X\right)-\text{min}\left(X\right)}\times 100\left(\text{forward standardization evaluation}\right).\\ g=\frac{\text{max}\left(X\right)-x}{\text{max}\left(X\right)-\text{min}\left(X\right)}\times 100\left(\text{inverse standardization evaluation}\right). \end{array}$$

In formula (8), x represents the original indicator data, g means the indicator score calculated after standardization, and X is the dataset of the indicators of all listed companies. Standardized evaluation retains the relationship of the original data and makes it dimensionless. Forward standardization is suitable for dealing with the indicators of “the bigger the better,” while inverse standardization is suitable for the opposite [23].

#### 3.2.2. Evaluation with Ranking Method

Considering the growth rate of operating income and net profit, the measurement standard should not be “the bigger the better.” For mature companies, their financial situation may be healthy, but the growth rate of operating income and net profit is relatively low compared with those companies in a growth period. Therefore, the ranking method is adopted in this research. By sorting these two indicators, the first place in the ranking is assigned 100 points, the last place in the ranking is assigned 0 points, and the middle-level companies are assigned equal and decreasing points so as to partially offset the phenomenon that the scores are too low or too concentrated caused by individual outliers [24]. The scoring criteria are shown in the following formula.

(9) $$\begin{array}{c} g_{rank}=100-\frac{100}{n}\cdot \left(rank-1\right). \end{array}$$

In formula (9), g_rank _ is the score after the ranking method, *n* is the total number of samples, and *rank* is the indicator ranking.

The article "Construction of a Fundamental Quantitative Evaluation Model of the A-Share Listed Companies Based on the BP Neural Network" was published in 2022. Journal: Comput Intell Neurosci.

#### 3.2.3. Evaluation by Moderate Analysis Method

Because companies need to ensure the appropriate ratio of assets and liabilities to cope with the debt repayment crisis and a certain leverage ratio to help themselves develop, the asset-liability ratio is generally considered to be more appropriate in the interval of (50% to 60%). Outside the interval, the more it deviates from the interval, the lower the score. The scoring criteria are shown in the following formula.

(10) $$\begin{array}{c} g_{lev}=\left\{\begin{array}{cc} 100, & 50\%\leq lev\leq 60\%\\ 100-5\cdot \left(lev-60\%\right)\times 100, & 60\%\leq lev\leq 80\%\\ 100-5\cdot \left(50\%-lev\right)\times 100, & 30\%\leq lev\leq 50\%\\ 0, & lev<30\%\;or\;lev>80\% \end{array}\right.. \end{array}$$

In formula (10), g_lev_ is the score of asset-liability ratio and *lev* is the asset-liability ratio of the company.

#### 3.2.4. Life Cycle Assessment

Listed companies have generally passed the start-up period. Because companies often adopt the expansion strategy in the growth period, their market share normally increases rapidly, and their organizational structure would be constantly improved [25], where the fundamental improvement expectation would be the highest. However, after the listed companies enter the mature stage, their market shares tend to be saturated, their organizational structure gradually matures, and their business activities remain in a stable stage [26]. At this time, the fundamentals of companies have entered a stable stage, and the expectation of their improvement is relatively weak. When companies run into a recession, their market share will be greatly reduced, their organizational structure will be redundant, and their fundamentals will gradually deteriorate. It can also be found that the allocation of fund companies is more inclined to companies in a growth stage. According to the cash flow portfolio method, the allocation ratios of Huaxia fund in the growth stage, mature stage, and recession stage are 54.41%, 28%, and 4.41%, respectively, which is similar to those of other fund companies [27]. Therefore, the expected fundamental improvement brought by the corporate life cycle is scored according to formula (11).

(11) $$\begin{array}{c} g_{T}=\left\{\begin{array}{c} 100,\;Growth\;Stage\\ 80,\;Mature\;Stage\\ 60,\;Recession\;Stage \end{array}\right.. \end{array}$$

In formula (11), *g*_*T*_ is the score given to the company according to the corporate life cycle theory.

### 3.3. Index Weight Calculation

In this paper, the annual report data of listed companies in 2020 are exported through Oriental Fortune Choice financial terminal, and some outliers are eliminated, where 3,096 samples are eventually obtained.

The article "Construction of a Fundamental Quantitative Evaluation Model of the A-Share Listed Companies Based on the BP Neural Network" was published in 2022. Journal: Comput Intell Neurosci.

Then, through the correlation coefficient formula (12), the correlation degree between the indicators is calculated. If the indicator correlation degree |*ρ*| > 0.8, then it is eliminated.  Table 3 shows the calculation result of the correlation coefficient of the indicators.

(12) $$\begin{array}{c} \left|\rho_{ij}\right|=\left|\frac{\text{COV}\left(X_{i},X_{j}\right)}{\sqrt{D\left(X_{i}\right)D\left(X_{j}\right)}}\right|,i=1\ldots 13,j=1\ldots 13\; \end{array}$$

As can be seen from the above table, the correlation between index X2 and index X9 is relatively high, the relatively rarely used total asset turnover rate (X9) is eliminated, and the current ratio (X2) is kept.

In the following part, the grey relational analysis will be adopted to calculate the initial weight and the expected output of the BP (back propagation) neural network.

Through the whole process of grey relational analysis shown in formulas (1) and (2), the results of the weight of each indicator are shown in Table 4. Using the weight and formula (3), the expected output can be obtained.

### 3.4. Construction of BP Neural Network

#### 3.4.1. Input Layer Neuron

According to Table 3, 13 secondary indicators such as asset-liability ratio, the growth rate of operating income, inventory turnover rate, and return on net assets are selected as input layer neurons based on the four dimensions of solvency, growth ability, operation ability, and profitability.

#### 3.4.2. Hidden Layer Neuron

The value range of the hidden layer node is calculated according to the empirical formula:

(13) $$\begin{array}{c} h=\sqrt{p+q}+a,\;a\in \left[1,10\right]. \end{array}$$

In formula (13), *h* represents the number of hidden layer nodes, *p* is the number of input layer neurons, and *q* is the number of output layer neurons. In this research, *p*=13 and *q*=1. The number of neurons of the hidden layer can be obtained in the range of [3,13].

#### 3.4.3. Output Layer Neuron

The number of output layer neurons is 1, which outputs the fundamental scores of listed companies with a value range of [0, 100]. The higher the output score, the better the fundamentals of the company.

*Determination of initial values of weights and thresholds.* In order to improve the learning speed of neural networks, the weights are set within the range of [0, 1] according to the usual practice, and random numbers in the range of [0, 1] are used as initial values of weights and thresholds.

### 3.5. Network Model Training

In the abovementioned 3,096 samples, 2,168 samples are randomly selected as training samples, which are recorded as TR_i_ (*i* = 1, 2,…, 2168), and the predicted value is obtained.

The article "Construction of a Fundamental Quantitative Evaluation Model of the A-Share Listed Companies Based on the BP Neural Network" was published in 2022. Journal: Comput Intell Neurosci.

Since the number of neurons of the hidden layer is in a certain interval, comparative experiments are conducted in order to optimize the parameter to obtain the smallest error. The results are shown in Figure 2.

From the figure, the conclusion is obvious that the smallest error can be gained when the number of neurons of the hidden layer is 10. Thus, the BP neural network designed in this paper sets the number of neurons in the input layer, hidden layer, and output layer as 13, 10, and 1, respectively. The structure of the BP neural network is shown in Figure 3. After 1000 times of training, the error is reduced to 1.01 × 10^−10^. According to the error trend chart in Figure 4, a quantitative evaluation model of the fundamentals of A-share listed companies in all industries.

A model based on BP neural network is established, and part of the training results of the BP neural network is shown in Table 5.

### 3.6. Simulation Result Analysis

It is necessary to test the network model in order to verify whether the BP neural network model is of the generalization ability. 604 samples are randomly selected from the remaining 1,208 samples and recorded as TE_j_ (*j* = 1, 2,…, 604) for testing, and the test results are shown in Table 6. The error distribution between training results and test results is shown in Figure 3.

According to Figure 5, the absolute errors of the training set and test set are mostly distributed in the interval of [-1.3 × 10^−5^, 9.6 × 10^−6^], where the errors are extremely small. Therefore, the BP neural network model designed in this paper is of good generalization ability and can be applied to the fundamental evaluation and analysis of A-share listed companies in all industries.

### 3.7. Robustness Test

In order to test the robustness of the model, this paper changes the evaluation interval of the asset-liability ratio from formula (10) to formula (14) as follows:

(14) $$\begin{array}{c} g_{lev}=\left\{\begin{array}{cc} 100, & 45\%\leq lev\leq 65\%\\ 100-5\cdot \left(lev-65\%\right)\times 100, & 65\%\leq lev\leq 80\%\\ 100-5\cdot \left(45\%-lev\right)\times 100, & 30\%\leq lev\leq 45\%\\ 0, & lev<30\%\;or\;lev>80\% \end{array}\right.. \end{array}$$

The new score is substituted into the model of the BP neural network, and the training error diagram shown in Figure 6 and the error distribution diagram shown in Figure 7 are obtained. It can be found that after 1000 iterations, the error is reduced to 2.0664 × 10^−8^, and the absolute errors are mostly distributed in [-4.6 × 10^−4^,3.6 × 10^−4^]. Therefore, the BP neural network model established in this paper is robust.

The article "Construction of a Fundamental Quantitative Evaluation Model of the A-Share Listed Companies Based on the BP Neural Network" was published in 2022. Journal: Comput Intell Neurosci.

## 4. Result Analysis

The author calculates the initial weight of each indicator of fundamental evaluation of listed companies through grey relational analysis and optimizes the weight through BP (back propagation) neural network. According to the calculation results of the training set data, the model can be established. According to the calculation results of the test set data, it can be concluded that the model has generalization ability. With this model, the fundamentals of A-share listed companies in China can be summarized to put forward some suggestions for fundamental evaluation.

### 4.1. Weight Analysis

The weights optimized by the BP neural network are shown in Table 7. Among them, solvency, growth ability, operation ability, profitability, and cycle judgment account for 29.61919%, 15.19587%, 14.02812%, 32.48885%, and 8.66757%, respectively. Profitability accounts for the highest proportion, followed by solvency, and there is little difference between growth ability and operational ability. It can be explained that profitability reflects the income quality of listed companies and is the most important part in the fundamental evaluation of listed companies. Solvency reflects the risk control of listed companies and is therefore of great significance in fundamental evaluation.

### 4.2. Scoring Results Analysis

The top 10 listed companies in the scoring order are selected on the basis of the scoring results, where it can be found in Table 8 that listed companies with higher scores have higher scores in return on net assets, quick ratio, and cash flow ratio. These three indicators reflect the efficiency of shareholders' funds, the solvency and liquidity of assets. Companies with good fundamentals have certain advantages in these aspects.

According to the descriptive statistics of each indicator shown in Table 9, China's listed companies have higher average scores in operating cost ratio and quick ratio, but lower scores in inventory turnover rate and accounts receivable turnover rate, which reflects that the listed companies have relatively strong profitability and solvency, while their operational ability is relatively weak. When making a stock selection, the important indicator of operational ability can be put into consideration to see if the company is leading in the industry.

## 5. Conclusion

This paper explores the application of BP (back propagation) neural networks in fundamental evaluation. Firstly, raw data of China's listed companies are imported and standardized by different scoring methods, which ensures rationality and comprehensiveness of the original score. Secondly, grey relational analysis is conducted in order to obtain the initial weight and expected output. Then, a 3-layer BP neural network is constructed after parameter optimization. The result is tested and validated. Finally, the result was analyzed from 2 aspects: weight analysis and scoring result analysis, where relative suggestions are provided for investors.

The article "Construction of a Fundamental Quantitative Evaluation Model of the A-Share Listed Companies Based on the BP Neural Network" was published in 2022. Journal: Comput Intell Neurosci.

Based on the experiment, a BP neural network used to evaluate the fundamentals of companies of all industries was constructed. This experiment proposed a new system of evaluation methods for all indicators that uses the important financial indexes of three statements for the first time. In addition, with the use of the corporate life cycle evaluation indicator, the companies with fundamental improvement expectations can be identified, which is an innovative attempt.

Although a BP neural network model has been constructed successfully, there are still some points that need to be improved.

1. The scores shown in Table 9 may not be rational since most of the samples seem to be in a recession stage, which disobeys common sense. Therefore, more precise algorithms should be applied to score the stage of companies.
2. There is still room for continued optimization in the internal structure of grey relational analysis and BP neural network, which can lead to more precise results.
3. Other advanced artificial neural networks can be used to compare with BP neural network, which is the direction of future efforts.

## Figures and Tables

**Figure 1:** The structure of the BP neural network.

**Figure 2:** Contrast of error under different parameter settings.

**Figure 3:** Structure diagram of BP neural network.

**Figure 4:** Training error diagram of BP neural network.

**Figure 5:** Error distribution diagram of BP neural network.

**Figure 6:** Training error diagram of robustness test.

**Figure 7:** Error distribution diagram of robustness test.

**Table 1:** Corporate life cycle judgment by the combination of cash flow components.

	Start-up	Growth	Mature	Recession			
Net cash flow from operating activities	−	+	+	−	+	+	−
Net cash flow from investment activities	−	−	−	−	+	+	+
Net cash flow from financing activities	+	+	−	−	+	−	−

**Table 2:** Selection of indicators.

Level 1 indicator	Level 2 indicator	Evaluation method	Symbol
Solvency	Asset-liability ratio	Moderate analysis method evaluation	X1
	Current ratio	Forward standardization evaluation	X2
	Quick ratio	Forward standardization evaluation	X3
	Cash flow ratio	Forward standardization evaluation	X4
Growth ability	Growth rate of operating income	Ranking method evaluation	X5
	Growth rate of net profit	Ranking method evaluation	X6
Operation ability	Inventory turnover rate	Forward standardization evaluation	X7
	Turnover rate of accounts receivable	Forward standardization evaluation	X8
	Turnover rate of total assets	Forward standardization evaluation	X9
Profitability	Return on net assets	Forward standardization evaluation	X10
	Net profit rate of sales	Forward standardization evaluation	X11
	Expense rate during sales period	Inverse standardization evaluation	X12
	Operating cost rate	Inverse standardization evaluation	X13
Periodic judgment	Corporate cycle judgment	Life cycle assessment	X14

The article "Construction of a Fundamental Quantitative Evaluation Model of the A-Share Listed Companies Based on the BP Neural Network" was published in 2022. Journal: Comput Intell Neurosci.

**Table 3:** Calculation result of correlation coefficient of indicators.

	X1	X2	X3	X4	X5	X6	X7	X8	X9	X10	X11	X12	X13	X14
X1	1.000	0.461	0.138	0.111	0.058	0.033	0.070	0.004	0.444	0.002	0.206	0.180	0.021	0.027
X2	0.461	1.000	0.176	0.080	0.043	0.031	0.018	0.064	0.947	0.041	0.277	0.354	0.062	0.012
X3	0.138	0.176	1.000	0.038	0.222	0.244	0.094	0.022	0.160	0.577	0.389	0.157	0.307	0.075
X4	0.111	0.080	0.038	1.000	0.238	0.145	0.361	0.312	0.064	0.195	0.218	0.070	0.279	0.049
X5	0.058	0.043	0.222	0.238	1.000	0.479	0.061	0.097	0.047	0.178	0.086	0.083	0.241	0.020
X6	0.033	0.031	0.244	0.145	0.479	1.000	0.027	0.054	0.035	0.247	0.105	0.084	0.127	0.012
X7	0.070	0.018	0.094	0.361	0.061	0.027	1.000	0.212	0.075	0.012	0.209	0.011	0.101	0.044
X8	0.004	0.064	0.022	0.312	0.097	0.054	0.212	1.000	0.050	0.075	0.086	0.146	0.055	0.053
X9	0.444	0.947	0.160	0.064	0.047	0.035	0.075	0.050	1.000	0.027	0.263	0.358	0.059	0.005
X10	0.002	0.041	0.577	0.195	0.178	0.247	0.012	0.075	0.027	1.000	0.192	0.092	0.286	0.082
X11	0.206	0.277	0.389	0.218	0.086	0.105	0.209	0.086	0.263	0.192	1.000	0.238	0.320	0.016
X12	0.180	0.354	0.157	0.070	0.083	0.084	0.011	0.146	0.358	0.092	0.238	1.000	0.016	0.138
X13	0.021	0.062	0.307	0.279	0.241	0.127	0.101	0.055	0.059	0.286	0.320	0.016	1.000	0.050
X14	0.027	0.012	0.075	0.049	0.020	0.012	0.044	0.053	0.005	0.082	0.016	0.138	0.050	1.000

**Table 4:** Calculation results of the weight of each indicator.

Level 1 indicator	Level 2 indicator	Symbol	Initial weight
Solvency	Asset-liability ratio	X1	6.79241
	Current ratio	X2	7.08412
	Quick ratio	X3	8.28635
	Cash flow ratio	X4	7.45493
Growth ability	Growth rate of operating income	X5	7.58143
	Growth rate of net profit	X6	7.61459
Operation ability	Inventory turnover rate	X7	7.04270
	Turnover rate of accounts receivable	X8	6.98549
Profitability	Return on net assets	X10	8.22696
	Net profit rate of sales	X11	7.75891
	Expense rate during sales period	X12	8.09567
	Operating cost rate	X13	8.41013
Periodic judgment	Corporate cycle judgment	X14	8.66630

**Table 5:** Part of training results of BP neural network.

Sample	Expected output	Actual output	Relative error (%)
TR1	53.73083	53.73004	0.00147
TR2	50.00218	50.00140	0.00157
TR3	46.79068	46.79015	0.00113
TR4	51.67963	51.67902	0.00119
TR5	33.12191	33.12213	0.00064
TR6	49.96475	49.96402	0.00145
TR7	53.76107	53.76060	0.00088
TR8	42.72477	42.72418	0.00138
TR9	44.14657	44.14600	0.00130
TR10	51.30777	51.30702	0.00146
TR11	47.05807	47.05735	0.00154
TR12	38.52720	38.52665	0.00144
TR13	49.56071	49.55982	0.00179
TR14	55.86725	55.86679	0.00083
TR15	48.76789	48.76711	0.00159
TR16	35.99980	36.00023	0.00119
TR17	61.00887	61.00867	0.00033
TR18	54.59437	54.59362	0.00137
TR19	48.13704	48.13696	0.00018
TR20	57.71973	57.71944	0.00052

The article "Construction of a Fundamental Quantitative Evaluation Model of the A-Share Listed Companies Based on the BP Neural Network" was published in 2022. Journal: Comput Intell Neurosci.

**Table 6:** Part of test results of BP neural network.

Sample	Expected output	Actual output	Relative error (%)
TE1	49.36534	49.36480	0.00109
TE2	58.05768	58.05710	0.00100
TE3	52.53170	52.53105	0.00125
TE4	44.80344	44.80370	0.00058
TE5	51.88164	51.88119	0.00087
TE6	47.13900	47.13851	0.00105
TE7	55.08644	55.08563	0.00147
TE8	62.44150	62.44073	0.00122
TE9	56.11946	56.11873	0.00129
TE10	44.80488	44.80430	0.00129
TE11	54.30785	54.30721	0.00118
TE12	56.28334	56.28285	0.00087
TE13	55.43343	55.43308	0.00064
TE14	53.17385	53.17326	0.00111
TE15	47.63893	47.63834	0.00124
TE16	45.67614	45.67584	0.00066
TE17	61.13550	61.13490	0.00098
TE18	55.73245	55.73178	0.00121
TE19	51.39826	51.39782	0.00084
TE20	55.22763	55.22727	0.00064

**Table 7:** Optimization results of the weight of each indicator.

Level 1 indicator	Level 2 indicator	Symbol	Initial weight	Optimized weight
Solvency	Asset-liability ratio	X1	6.79241	6.79240
	Current ratio	X2	7.08412	7.08433
	Quick ratio	X3	8.28635	8.28747
	Cash flow ratio	X4	7.45493	7.45499
Growth ability	Growth rate of operating income	X5	7.58143	7.58136
	Growth rate of net profit	X6	7.61459	7.61451
Operation ability	Inventory turnover rate	X7	7.04270	7.04273
	Turnover rate of accounts receivable	X8	6.98549	6.98539
Profitability	Return on net assets	X10	8.22696	8.22687
	Net profit rate of sales	X11	7.75891	7.75800
	Expense rate during sales period	X12	8.09567	8.09591
	Operating cost rate	X13	8.41013	8.40807
Periodic judgment	Corporate cycle judgment	X14	8.66630	8.66757

**Table 8:** Scores of each indicator of the 10 listed companies with the highest scores.

Sample	X1	X2	X3	X4	X5	X6	X7	X8	X10	X11	X12	X13	X14	Score
S1	100.000	34.503	100.000	100.000	15.700	34.400	100.000	100.000	100.000	81.108	67.500	100.000	60.000	76.410
S2	42.100	100.000	100.000	100.000	88.300	2.800	100.000	95.177	100.000	81.296	0.000	100.000	60.000	74.428
S3	72.250	70.000	92.482	100.000	28.400	13.100	85.031	100.000	89.890	50.455	81.165	76.081	100.000	74.056
S4	24.700	100.000	100.000	100.000	77.500	83.500	0.000	100.000	100.000	100.000	100.000	0.000	60.000	73.005
S5	67.950	55.135	81.812	100.000	62.700	75.000	58.710	100.000	100.000	83.214	0.000	69.767	60.000	70.090
S6	0.000	19.434	94.273	100.000	74.900	91.800	38.377	100.000	88.921	61.046	68.471	92.643	60.000	69.586
S7	100.000	7.715	90.124	100.000	31.000	60.100	84.081	20.917	73.218	66.218	59.180	98.857	100.000	69.504
S8	100.000	46.341	100.000	97.727	19.800	25.200	75.463	68.541	100.000	65.569	100.000	43.964	60.000	69.478
S9	80.250	18.387	91.789	100.000	10.100	47.100	100.000	100.000	93.759	66.331	32.890	100.000	60.000	69.326
S10	77.350	13.430	88.656	51.429	93.200	88.600	100.000	9.622	87.519	59.887	69.430	80.162	60.000	68.322

The article "Construction of a Fundamental Quantitative Evaluation Model of the A-Share Listed Companies Based on the BP Neural Network" was published in 2022. Journal: Comput Intell Neurosci.

**Table 9:** Descriptive statistics of scores of all indicators.

	X1	X2	X3	X4	X5	X6	X7	X8	X10	X11	X12	X13	X14	Score
Max	0.000	0.000	0.000	0.000	0.000	0.000	0.000	0.000	0.000	0.000	0.000	0.000	60.000	18.372
Min	100.000	100.000	100.000	100.000	100.000	100.000	100.000	100.000	100.000	100.000	100.000	100.000	100.000	76.410
Average	43.854	22.074	68.523	30.535	49.972	49.972	21.364	20.933	65.064	47.595	61.820	74.441	64.289	48.940

## Data Availability

The data used to support the findings of this study are available from the corresponding author upon request.
